The article "FXYD6 Regulates Chemosensitivity by Mediating the Expression of Na+/K+-ATPase α1 and Affecting Cell Autophagy and Apoptosis in Colorectal Cancer" was retracted in 2024. Reasons: signs of a paper mill; compromised peer review; unreliable results or conclusions.

# FXYD6 Regulates Chemosensitivity by Mediating the Expression of Na+/K+-ATPase *α*1 and Affecting Cell Autophagy and Apoptosis in Colorectal Cancer

**DOI:** 10.1155/2021/9986376

**Published:** 2021-06-09

**Authors:** Wen Luo, Qingan Liu, Xinwen Chen, Haijun Liu, Bin Quan, Jinli Lu, Ke Zhang, Xiangling Wang

**Affiliations:** Department of General Surgery, Changde First People's Hospital, Changde, Hunan 415000, China

## Abstract

**Purpose:**

Chemoresistance is a challenge of improving chemotherapeutic efficacy and prolonging survival time for patients with colorectal cancer (CRC); it is the major cause of frequent recurrence, rapid metastasis, and poor prognosis for CRC patients. FXYD6 is a regulator of Na+/K+-ATPase which is depressed in chemoresistant CRC patients. However, the biological roles of FXYD6 on regulating chemoresistance in CRC are still unclear.

**Methods:**

GSE3964 and GSE69657 from GEO DataSets were used to analyze the relationship of genes and chemoresistance. The FXYD6 expression level was detected by western blotting and real-time PCR and also analyzed from TCGA DataSet. To investigate the functional role of FXYD6 and ATP-*α*1, FXYD6 and ATP-*α*1 functional cell models were constructed. Drug sensitivity and cell proliferation were performed by MTT assay. Autophagy and apoptosis were conducted by autophagy fluorescence analysis and flow cytometric analysis, respectively. Autophagy and apoptosis markers were tested by western blotting.

**Results:**

FXYD6 was downregulated in CRC resistant patients and irinotecan- (Iri-) resistant SW620 cells (SW620/Iri). FXYD6 silence inhibited cell apoptosis and enhanced prosurvival autophagy, whereas FXYD6 overexpression produced the opposite effect which alleviated the drug resistance to irinotecan and oxaliplatin of CRC cells. FXYD6 regulates chemosensitivity by mediating the expression of Na+/K+-ATPase *α*1 and affecting cell autophagy and apoptosis in colorectal cancer.

**Conclusion:**

FXYD6 functions as a chemosensitivity regulator which may predict the curative effect of chemotherapy in colorectal cancer.

## 1. Introduction

Colorectal cancer (CRC) accounts for approximately 10% of all annually diagnosed cancers and cancer-related deaths globally and is the world's fourth most deadly cancer [1]. The treatment methods for CRC include surgical excision, chemotherapy, radiotherapy, and the recent application of molecularly targeted therapy and immunotherapy. However, chemotherapy is regarded as the standard mode of treatment for CRC patients [2], particularly those with advanced tumors. Iri is a camptothecin derivative and a prodrug comprising the active metabolite SN-80, which inhibits the activity of eukaryotic type IB topoisomerases (Top1) and promotes cancer cell death [3]. Presently, Iri is always used in combination with oxaliplatin (Oxa), 5-fluorouracil (5-FU), and another molecularly targeted anticancer drug, resulting in a significantly prolonged survival time [4]. Oxa is a third-generation platinum drug that induces apoptotic cell death and prolongs the G2 phase cell cycle arrest by covalently binding to DNA and forming platinum-DNA adducts [5]. Capecitabine, a prodrug of 5-FU, is another fluorouracil antimetabolite used frequently in CRC [6]. Although these chemotherapeutic drugs are usually used as first-line treatment and have an obvious effect on CRC, the majority of patients finally develop resistance, resulting in poor drug efficacy and prognosis [7, 8]. Thus, the mechanisms of chemoresistance in CRC patients should be illustrated.

The article "FXYD6 Regulates Chemosensitivity by Mediating the Expression of Na+/K+-ATPase α1 and Affecting Cell Autophagy and Apoptosis in Colorectal Cancer" was retracted in 2024. Reasons: signs of a paper mill; compromised peer review; unreliable results or conclusions.

FXYD proteins belong to a family of small membrane proteins. They are auxiliary subunits and function as regulators of Na+/K+-ATPase [9], such as FXYD domain-containing ion transport regulator 6 (FXYD6) [10]. Dysregulation of FXYD6 results in the development of multiple cancers. Some studies have reported that FXYD6 is highly expressed in cholangiocarcinoma [11] and hepatocellular carcinoma [12]; alternatively, the inhibition of this protein has been demonstrated in thyroid carcinoma [13]. FXYD6 is positively associated with chemotherapy sensitivity in CRC [14]. Nonetheless, the molecular mechanism involved has not been extensively studied so far.

Na+/K+-ATPase is a member of the P-type ATPase superfamily, and its functions mainly include pumping ions across the cell membrane to maintain ionic and osmotic balance and conducting intracellular signals [15]. As a signal transducer, Na+/K+-ATPase mediates various intracellular signaling pathways such as the PI3K/Akt/mTOR and the Src-EGFR-Ras-Raf-kinase pathway, which regulates tumor cell proliferation and survival [15, 16]. Besides, Na+/K+-ATPase was directly connected to Bcl-2 and thereby involved in regulating both cell survival and apoptosis [17]. Na+/K+-ATPase is related to cancer development and progression and is a target for anticancer treatment [18]. The expression level of Na+/K+-ATPase relates to chemoresistance and multidrug resistance (MDR) in cancer cells; Na+/K+-ATPase expression is downregulated in MDR cells compared with sensitive cells [19]. Moreover, the inhibition of Na+/K+-ATPase leads to an increase in the mRNA expression of MDR1 [20]. In other words, Na+/K+-ATPase is an important target for anticancer treatment. It acts as a key cause of chemoresistance.

Autophagy is a conserved catabolic process and essential for maintaining homeostasis. Furthermore, autophagy plays a significant role in cell survival and maintenance through the degradation of the cytoplasmic organelles, proteins, and macromolecules and the recycling of the breakdown products [21]. The process of autophagy can be promoted by cellular stress, such as starvation, hypoxia, inflammation, and the use of anticancer drugs [22, 23], which can prevent cell damage, promote cell survival under conditions of nutrient deficiency, and respond to cytotoxic stimuli [24]. Autophagy induced by anticancer drugs can protect MDR cancer cells from chemotherapy. The primary mechanism of MDR is the overexpression of ATP-binding cassette transporters to promote drug influx and cause a decrease in intracellular drug concentration [25]. In the present study, the role of FXYD6 in chemosensitivity was investigated and it was found that FXYD6 was decreased in CRC chemoresistance patient tissues when compared with CRC sensitive patients. FXYD6 modulated CRC chemosensitivity through mediating the expression of ATP-*α*1, which affected both cell autophagy and apoptosis in CRC.

The article "FXYD6 Regulates Chemosensitivity by Mediating the Expression of Na+/K+-ATPase α1 and Affecting Cell Autophagy and Apoptosis in Colorectal Cancer" was retracted in 2024. Reasons: signs of a paper mill; compromised peer review; unreliable results or conclusions.

## 2. Materials and Methods

### 2.1. Clinical Cancer Samples and Cell Lines

All samples were obtained from Changde First People's Hospital, Hunan, China, and samples were stored at -80°C until used. This study was approved by the Medical Ethics Committee of Changde First People's Hospital, acting as the Institutional Review Board (Number: 2020-098-01). Five CRC patients who were not treated with chemotherapeutic drugs before surgery were recruited (Table 1).

The human colorectal cancer cell lines HCT116, LOVO, SW480, and SW620 and normal cell line HCoEpic were purchased from the American Type Culture Collection (ATCC, Manassas, VA, USA) and cultured in the RPMI-1640 medium (Gibco, Rockville, MD, USA) supplemented with 10% fetal bovine serum (FBS, Life Technologies, Carlsbad, CA, USA) and 1% penicillin and streptomycin sulfate (Solarbio, Beijing, China). Cells were incubated at 37°C with 5% CO_2_.

### 2.2. Online Data Acquisition

To find the genes associated with chemoresistance in CRC, GSE3964, including sensitive and resistant patients treated with Iri, and GSE69657, including sensitive and resistant patients treated with Oxa, were used. The sensitive patients were used as the control group, and differential analysis of drug-resistant genes was carried out between the sensitive group and the resistant group. Morpheus software was used for cluster analysis of mRNA between the sensitive group and the resistant group with the most significant difference for two raw datasets. ∣log2FC | >1 and *P* < 0.05 were used as selection conditions for differentially expressed genes. Besides, the normalized RNA-seq data from the CRC dataset were downloaded from The Cancer Genome Atlas (TCGA) DataSet.

The article "FXYD6 Regulates Chemosensitivity by Mediating the Expression of Na+/K+-ATPase α1 and Affecting Cell Autophagy and Apoptosis in Colorectal Cancer" was retracted in 2024. Reasons: signs of a paper mill; compromised peer review; unreliable results or conclusions.

### 2.3. Chemotherapeutic Drug-Resistant Cell Line Construction

The SW620 cells with low Iri sensitivity titled SW620/Iri were selected from the wild-type SW620 cell line; the construction method was referred to published paper [26]. SW620 cells were seeded on a 12-well plate (3 × 10^5^ cells per well) and incubated in a medium containing Iri (Selleck, Shanghai, China) at an initial concentration of 2 *μ*M until the cells grew stably. Subsequently, Iri concentration was gradually increased until cells can grow well at 10 *μ*M. Then, the SW620/Iri cell line which can tolerate 10 *μ*M Iri was obtained successfully.

### 2.4. Real-Time PCR (RT-PCR)

Total RNAs were extracted from cancer samples and cultured cells with TRIzol (TaKaRa, Tokyo, Japan). mRNA was reverse-transcribed with a PrimeScript RT Reagent Kit (TaKaRa, Japan) to cDNA. GAPDH was used as the normalization control for FXYD6 and ATP-*α*1. Primer pair sequences are listed in Table 2. cDNA was mixed with SuperReal PreMix Plus (SYBR Green) kits (Tiangen, Beijing, China) and each primer pair to produce a 20 *μ*L reaction mixture. All RT-PCR tests were conducted with an ABI 7500 RT-PCR system (Applied Biosystems, Carlsbad, CA, USA). The thermocycling conditions were as follows: initial denaturation at 95°C for 15 min and 45 cycles of 95°C for 10 sec, 60°C for 20 sec, and 72°C for 60 sec. Each reaction was done in triplicate, and the average 2^-*ΔΔ*Ct^ was used in data analysis.

### 2.5. Plasmid Transfections

The overexpressed vectors and small interfering RNA (siRNA) were both obtained from GenePharma (Shanghai, China), containing the FXYD6 and ATP-*α*1 overexpressed vectors pcDNA3.1-FXYD6 (FXYD6) and pcDNA3.1-ATP-*α*1 (ATP-*α*1) and the empty vector pcDNA3.1 (control), as well as siRNA against FXYD6 (siFXYD6) and ATP-*α*1 (siATP-*α*1) and the negative control siRNA (siNC). The interference sequences are listed in Table 3. Plasmids and siRNA were transfected using Lipofectamine 3000 (Invitrogen, Carlsbad, CA, USA) according to the manufacturer's protocols.

### 2.6. Drug Sensitivity Assays

3-(4,5-Dimethylthiazol-2-yl)-2,5-diphenyltetrazolium bromide (MTT) assays were carried out in the FXYD6 silenced SW620 cells and the FXYD6 overexpressed SW620/Iri cells to confirm the drug concentration of Iri and Oxa (Selleck, Shanghai, China). Cells were seeded on 96-well plates (5 × 10^3^ cells per well) and incubated overnight in a 0.2 mL fresh medium. Then, cells were exposed to different doses of Iri and Oxa, respectively, for 24 h. After reacting with 20 *μ*L 5 mg/mL MTT (Sigma, St. Louis, MO, USA) at 37°C for 4 h, the culture medium was removed and 150 *μ*L dimethylsulfoxide (DMSO) was added. The reactions were performed in triplicate, and absorbance was measured at 490 nm using an enzyme-linked immunosorbent assay reader (BioTek, Vermont, VT, USA).

The article "FXYD6 Regulates Chemosensitivity by Mediating the Expression of Na+/K+-ATPase α1 and Affecting Cell Autophagy and Apoptosis in Colorectal Cancer" was retracted in 2024. Reasons: signs of a paper mill; compromised peer review; unreliable results or conclusions.

### 2.7. Cell Proliferation Assays

Cells were seeded on 96-well plates (5 × 10^3^ cells per well) and incubated overnight in a 0.2 mL fresh medium. Subsequently, cells were, respectively, pretreated with the autophagic inhibitor 3-methyladenine (3-MA) and autophagic stimulator rapamycin (Rapa) for 48 h; DMSO and PBS were used as the control. Then, cells were exposed to 10 *μ*M Iri and 0.5 *μ*M Oxa, respectively. MTT assays were performed to evaluate cell proliferation at 0 h, 24 h, 48 h, 72 h, and 96 h.

To research the influence of FXYD6 and ATP-*α*1 on cell proliferation, cells were exposed to 10 *μ*M Iri and 0.5 *μ*M Oxa, respectively. MTT assays were conducted, respectively, at 0 h, 24 h, 48 h, 72 h, and 96 h to evaluate cell proliferation.

The reactions were performed in triplicate, and average optical density (OD) was used to calculate the cell survival rate. The cell survival rate was calculated according to the following formula: cell survival rate = (mean OD of treated wells/mean OD of control wells) × 100%.

### 2.8. Cell Apoptosis Analysis

The FITC Annexin V Apoptosis Detection Kit (KeyGen Biotech, Nanjing, China) was used according to the manufacturer's protocol. Treated SW620 and SW620/Iri cells were collected and suspended in an annexin-binding buffer. Then, cells were stained with FITC Annexin V and propidium iodide (PI). Flow cytometry was conducted on FACScan flow cytometry (BD Biosciences, San Jose, CA, USA).

### 2.9. Autophagy Fluorescence Analysis

Cells were plated in 6-well plates and incubated for 48 h after transfection. The tandem fluorescent mRFP-GFP-LC3 plasmid was obtained from GenePharma Biotechnology (Suzhou, China). Autophagic changes were observed under a fluorescence microscope (E3I-630, MOTIC, USA) that visualized 200x images. The numbers of red fluorescent protein (RFP) puncta (red puncta) were used to evaluate the activity of autophagy.

### 2.10. Western Blotting

Cell proteins were lysed in a RIPA lysis buffer (Solarbio, Beijing, China) with a proteinase inhibitor cocktail (Roche, Mannheim, Germany). Samples were separated by 12% SDS-PAGE and transferred to nitrocellulose membranes (Hybond, Amersham Pharmacia Biotech, Piscataway, NJ, USA). The membranes were blocked for 1 h at room temperature with 3% nonfat milk/TBST and subsequently incubated in the primary antibodies anti-FXYD6, anti-ATP-*α*1, anti-LC3II/I, anti-P62, anti-Beclin1, anti-BAX, anti-Bcl-2, or anti-*β*-actin for 2 h at room temperature and washed 3 times in TBST. *β*-Actin was used as the internal control. Antibody information are shown in Table 4. Then, the membranes were incubated in the secondary antibody for 2 h at room temperature conjugated to horseradish peroxidase. The signals were detected by enhanced chemiluminescence (NEN, Boston, MA, USA).

The article "FXYD6 Regulates Chemosensitivity by Mediating the Expression of Na+/K+-ATPase α1 and Affecting Cell Autophagy and Apoptosis in Colorectal Cancer" was retracted in 2024. Reasons: signs of a paper mill; compromised peer review; unreliable results or conclusions.

### 2.11. Statistical Analysis

Data were expressed as means ± SD; the statistical differences were analyzed by Student's *t*-test and analysis of variance (ANOVA). Statistical probability (*P*) in figures and figure legends were expressed as follows: ^∗^*P* < 0.05, ^∗∗^*P* < 0.01, and ^∗∗∗^*P* < 0.001.

## 3. Results

### 3.1. FXYD6 Was Depressed in Chemoresistant Colorectal Cancer and Related to Chemoresistance

To investigate the genes related to chemoresistance in CRC, we performed an analysis of mRNA expression data which was downloaded from GEO DataSets (GSE3964 and GSE69657). The result of data analysis showed that FXYD6 was reduced obviously in the resistant group (R) compared to the sensitive group (S), which suggested that the lower expression level of FXYD6 was positively correlated to Iri and Oxa resistance in CRC (Figure 1(a)). To understand FXYD6 expression in CRC, we firstly analyzed the data including 41 normal tissue samples and 286 primary tumor tissue samples from TCGA; the expression levels of FXYD6 in tumor samples were observably decreased (Figure 1(b)). Then, FXYD6 expression was measured in five clinically matched CRC tissue samples and adjacent tissue samples by RT-PCR; the result also indicated that FXYD6 was decreased in CRC (Figure 1(c)).

Compared to HCoEpic, FXYD6 was downregulated in HCT116 and SW620 cells when tested using RT-PCR (Figure 1(d)), while in HCT116, SW480, and SW620 cells by western blotting (Figure 1(e)). Finally, the SW620 cell line with the lower expression of FXYD6 was used in this study. To observe the expression of FXYD6 in chemoresistant cells, the FXYD6 expression was compared in SW620 and its resistant cell line SW620/Iri. It was found that FXYD6 was inhibited in SW620/Iri (Figures 1(f) and 1(g)).

### 3.2. FXYD6 Regulated Chemosensitivity through Mediating Apoptosis of CRC Cells

To clarify the effect of FXYD6 overexpression and underexpression on cells exposed to Oxa and Iri, the FXYD6 loss-of-function cell model was successfully constructed by transfecting the siRNA-FXYD6 (siFXYD6) into SW620 cells; and the FXYD6 gain-of-function cell model was successfully constructed by transfecting the FXYD6 overexpressed plasmid (FXYD6) into SW620/Iri cells (Figure 2(a)). Then, FXYD6 silenced SW620 cells and SW620/Iri-FXYD6 overexpressed cells were, respectively, exposed in different Iri and Oxa to confirm the drug concentration when the cell proliferation rate changed significantly compared to the non-drug-treated group. When cells were treated with 10 *μ*M Iri and 0.5 *μ*M Oxa, the cell survival rate was significantly decreased (Figure 2(b)). In the following drug treatment, 10 *μ*M Iri and 0.5 *μ*M Oxa were used. To further explore the effect of FXYD6 expressed to cell apoptosis induced by Oxa and Iri, the cell apoptosis was observed using flow cytometric analysis in SW620-FXYD6 silenced cells and SW620/Iri-FXYD6 overexpressed cells which were, respectively, exposed at 10 *μ*M Iri and 0.5 *μ*M Oxa. Early apoptosis (LR) and late apoptosis (UR) were used to analyze the apoptosis rate. It was found that cell apoptosis was significantly increased when FXYD6 was overexpressed but significantly decreased when FXYD6 was silenced (Figure 2(c)). To examine whether the apoptosis elements such as Bcl-2 and BAX were involved in chemoresistance regulated by FXYD6, we analyzed the expression of Bcl-2 and BAX in FXYD6 silenced SW620 cells and FXYD6 overexpressed SW620/Iri cells. The results showed that increased Bcl-2 expression and decreased BAX expression were detected when FXYD6 was silenced, which suggested that cell apoptosis was inhibited (Figure 2(d)). All these data indicated that the low expression level of FXYD6 was related to suppressive cell apoptosis which led to irinotecan and oxaliplatin resistance in CRC.

The article "FXYD6 Regulates Chemosensitivity by Mediating the Expression of Na+/K+-ATPase α1 and Affecting Cell Autophagy and Apoptosis in Colorectal Cancer" was retracted in 2024. Reasons: signs of a paper mill; compromised peer review; unreliable results or conclusions.

### 3.3. FXYD6 Regulated Chemoresistance through Mediating CRC Cell Autophagy

We hypothesized that FXYD6 was involved in chemosensitivity through mediating CRC cell autophagy. To verify this hypothesis, autophagy fluorescence analysis was performed. mRFP-GFP-LC3 and FXYD6 plasmids were cotransfected into SW620/Iri cells, mRFP-GFP-LC3 and siFXYD6 were cotransfected into SW620 cells, and cells were, respectively, exposed at 10 *μ*M Iri and 0.5 *μ*M Oxa. It was observed that fewer autophagosomes (red puncta) were generated when FXYD6 was upregulated, while more autophagosomes were shown when FXYD6 was downregulated (Figure 3(a)). Western blotting revealed a consistent result; decreased LC3II/I and Beclin1 and increased P62 were shown when FDYD6 was overexpressed, while increased LC3II/I and Beciln 1 and decreased P62 were shown when FXYD6 was underexpressed, which suggested that autophagy was promoted when FXYD6 was silenced and inhibited when FDYD6 was overexpressed (Figure 3(b)). FXYD6 regulating Iri and Oxa sensitivity through mediating CRC cell autophagy was verified. Using MTT assays, it was observed that the cell survival rate was obviously enhanced in FXYD6 overexpressed SW620/Iri cells treated with Rapa, while the cell survival rate was much lower in FXYD6 silenced SW620 cells treated with 3-MA when compared with the DMSO group, which revealed that apoptosis was enhanced through inhibiting prosurvival autophagy (Figure 3(c)). These results were confirmed by flow cytometric analysis; early apoptosis (LR) and late apoptosis (UR) were used to analyze the apoptosis rate. Decreased apoptosis was shown under Rapa treatment, while increased apoptosis was shown under 3-MA treatment (Figure 3(d)). In brief, the underexpression of FXYD6 caused decreased apoptosis by activating prosurvival autophagy, so CRC cells became less sensitive to chemodrugs.

The article "FXYD6 Regulates Chemosensitivity by Mediating the Expression of Na+/K+-ATPase α1 and Affecting Cell Autophagy and Apoptosis in Colorectal Cancer" was retracted in 2024. Reasons: signs of a paper mill; compromised peer review; unreliable results or conclusions.

### 3.4. FXYD6 Regulated Cell Apoptosis and Autophagy by Mediating the Activity of ATP-*α*1 in Chemosensitivity Regulation

The ATP-*α*1 subunit is essentially omnipresent at the tissue and cellular levels [27]. Firstly, the expression level of ATP-*α*1 in SW620 and SW620/Iri cells was tested using western blotting and RT-PCR. It was found that the expression of ATP-*α*1 was significantly decreased in SW620/Iri cells (Figure 4(a)), which indicated that depressed ATP-*α*1 facilitated Iri resistance. Next, FXYD6 and ATP-*α*1 were silenced and enhanced, respectively, in SW620/Iri and parental cells for researching the relationship between FXYD6 and ATP-*α*1. Western blotting showed that ATP-*α*1 was decreased following FXYD6 knockdown and increased following FXYD6 overexpression, while FXYD6 expression had no obvious change when ATP-*α*1 was downregulated or upregulated (Figure 4(b)). These results suggested that ATP-*α*1 was one of the downstream targets of FXYD6. To verify that ATP-*α*1 was a bridge factor for FXYD6 to regulate apoptosis and autophagy, FXYD6 silenced SW620 cells were transfected with the ATP-*α*1 overexpressed plasmid, while FXYD6 overexpressed SW620/Iri cells were transfected with the siATP-*α*1 for 48 h, and cells were treated with 10 *μ*M Iri and 0.5 *μ*M Oxa (Figure 4(c)). Apoptosis and autophagy elements were detected by western blotting. When ATP-*α*1 was upregulated in FXYD6 silenced SW620 cells, compared with FXYD6 silenced SW620 cells without ATP-*α*1 overexpression, decreased LC3II/I and increased P62, as well as increased BAX and decreased Bcl-2, were shown which indicated that prosurvival autophagy was inhibited and apoptosis was promoted obviously; when ATP-*α*1 was silenced in FXYD6 overexpressed SW620/Iri cells, compared with FXYD6 overexpressed SW620/Iri cells without ATP-*α*1 silence, increased LC3II/I and decreased P62, as well as decreased BAX and increased Bcl-2, were tested which indicated that autophagy was enhanced again and apoptosis was inhibited to some extent (Figure 4(d)). MTT assays produced consistent results; the cell survival rate was significantly higher in FXYD6 overexpressed cells with ATP-*α*1 silence when compared with FXYD6 overexpressed SW620/Iri cells without ATP-*α*1 silence (red solid line and blue dotted line), while the cell survival rate was significantly lower in FXYD6 silenced cells with ATP-*α*1 overexpression when compared with FXYD6 silenced SW620/Iri cells without ATP-*α*1 overexpression (red dotted line and blue solid line) (Figure 4(e)). Autophagy fluorescence analysis clearly showed that the autophagy was inhibited in FXYD6 silenced SW620 cells with ATP-*α*1 overexpression but enhanced in FXYD6 overexpressed SW620/Iri cells with ATP-*α*1 knockdown (Figure 4(f)). Cell apoptosis analysis obviously revealed that the apoptosis was enhanced in FXYD6 silenced SW620 cells with ATP-*α*1 overexpression but weakened when ATP-*α*1 was silenced in FXYD6 overexpressed SW620/Iri cells (Figure 4(g)). These results indicated that the regulation of FXYD6 on cell viability and autophagy was mediated by ATP-*α*1 to some extent.

The article "FXYD6 Regulates Chemosensitivity by Mediating the Expression of Na+/K+-ATPase α1 and Affecting Cell Autophagy and Apoptosis in Colorectal Cancer" was retracted in 2024. Reasons: signs of a paper mill; compromised peer review; unreliable results or conclusions.

## 4. Discussion

Chemotherapy regimens containing Iri or Oxa have been effectively used as first-line or adjuvant treatment after surgical debulking in CRC patients [28–31]. However, frequent recurrence, rapid metastasis, and poor prognosis generally occur following the development of drug resistance. The use of molecularly targeted drugs must be confirmed if the patient is eligible for drugs; however, it is beneficial for only a portion of the CRC patients who carry the drug-sensitive gene [32–34]. Despite the presence of several biomarkers, responses to novel immunotherapy are unsatisfactory in CRC patients [35–38]. Conventional chemotherapy continues to remain the first choice of treatment for CRC.

Na+/K+-ATPase is expressed as four *α* isoforms, three *β* isoforms, and seven FXYD subunit isoforms [27]. The *α*1 and *β*1 isoforms are expressed in CRC; some studies report that the ATP-*α*1 subunit is involved in autophagy and apoptosis, whereas the role of the *β*1 subunit is unclear [39, 40]. The expression levels of the Na+/K+-ATPase isoforms vary in different types of cancer. The ATP-*α*1 subunit is upregulated in non-small-cell lung cancer, renal cell carcinoma, glioma, and melanoma and downregulated in prostate cancer [18]. Additionally, the ATP-*α*1 subunit is downregulated, and the Na+/K+-ATPase *α*3 (ATP-*α*3) subunit is upregulated in colon carcinoma [41]. In the present study, ATP-*α*1 was downregulated in SW620/Iri cells compared with SW620 cells, which could cause an increase in drug resistance. ATP-*α*3 was upregulated in colon cancer; however, the role of FXYD6 in modulating the expression of ATP-*α*3 and regulating cell autophagy and apoptosis leading to drug sensitivity needs to be investigated in the future. Na+/K+-ATPase can circumvent various resistance pathways, including the MDR pathway, by regulating the expression of MDR-related genes to induce chemoresistance [42]. In SW620/Iri cells, if the underexpression of ATP-*α*1 can lead to an increase in the expression of MDR, resulting in drug resistance, the expression level of MDR-related genes will be explored clearly.

The article "FXYD6 Regulates Chemosensitivity by Mediating the Expression of Na+/K+-ATPase α1 and Affecting Cell Autophagy and Apoptosis in Colorectal Cancer" was retracted in 2024. Reasons: signs of a paper mill; compromised peer review; unreliable results or conclusions.

FXYD6 expression is upregulated [11, 12] or downregulated [13] in several cancers. There is no clear evidence to confirm that FXYD6 acts as a tumor suppressor. A few studies have reported that FXYD6 is upregulated in colon cancer [12]. Significantly high levels of FXYD6 were detected in cancerous tissues (17/17) when compared with the corresponding normal tissues (4/6). An analysis of TCGA data, which contained 286 primary CRC tumors and normal tissues, demonstrated that FXYD6 was silenced in CRC. Furthermore, we verified that FXYD6 was silenced in CRC resistant patients by analyzing the public data from the GEO DataSets and testing the expression level of the protein in SW620/Iri cells. Upregulating the expression level of FXYD6 showed that CRC cells are sensitive to Iri and Oxa. Consistent with the results of a previous study [14], the expression level of FXYD6 was positively correlated with chemotherapy sensitivity in the present study. Additionally, FXYD6 was reported to form a panel in combination with another six genes to predict early relapse in thyroid cancer [43]. These findings indicate that FXYD6 might prove to be a promising indicator of the risk of recurrence in CRC.

FXYD6 expression levels were lower in CRC patients when compared with normal individuals, as demonstrated in TCGA data analysis. Furthermore, FXYD6 was underexpressed in four out of five matched CRC tissues that were tested for FXYD6 expression. This low expression of FXYD6 might have resulted in the drug resistance to Iri and Oxa before the CRC patient will be treated by chemotherapy, given that the expression level of FXYD6 has been known. To obtain a good treatment outcome, we believe that patients with low expression levels of FXYD6 should not receive chemotherapy regimens containing Iri and Oxa. Hence, the level of FXYD6 expression in the patients should be determined to optimize the chemotherapeutic strategy.

## 5. Conclusion

In the present study, FXYD6 expression was lower in CRC patients who were resistant to Iri and Oxa. FXYD6 knockdown resulted in a decrease in the ATP-*α*1 expression; additionally, cell apoptosis was inhibited and cell prosurvival autophagy was enhanced; consequently, the CRC cells were less sensitive to Iri and Oxa. Conversely, upregulation of FXYD6 made the CRC cells more sensitive to Iri and Oxa. Our findings indicate that FXYD6 functions as a regulator of chemosensitivity and may predict the curative effect of chemotherapy in CRC.

The article "FXYD6 Regulates Chemosensitivity by Mediating the Expression of Na+/K+-ATPase α1 and Affecting Cell Autophagy and Apoptosis in Colorectal Cancer" was retracted in 2024. Reasons: signs of a paper mill; compromised peer review; unreliable results or conclusions.

## Figures and Tables

**Figure 1:** FXYD6 was silenced in chemoresistance colorectal cancer and related to chemosensitivity. (a) FXYD6 expression was analyzed in the resistant and sensitive groups treated by Oxa or Iri from GSE69657 and GSE3964. The green box and orange box indicated the resistant group (R) and sensitive group (S), respectively. (b) Statistical analysis of FXYD6 expression data in CRC from TCGA DataSet; the purple box indicated the normal tissue sample; the red box indicated the primary tumor tissue sample. (c) FXYD6 expression was measured in cancer tissues and relative adjacent tissues from five CRC patients by RT-PCR. (d) Expression of FXYD6 was detected by RT-PCR in the different CRC cell lines and normal cell line HCoEpic. (e) The upper panel showed the western blotting of FXYD6 in the different CRC cell lines and normal cell line HCoEpic; *β*-actin was used as the internal control. The lower panel was the quantification of FXYD6 by the ImageJ program. (f) FXYD6 expression was tested in CRC cell lines SW620 and SW620/Iri by RT-PCR. (g) The left panel showed the protein levels of FXYD6 in SW620 and SW620/Iri cells by western blotting; *β*-actin was used as the internal control. The right panel was the quantification of FXYD6 by the ImageJ program.

**Figure 2:** FXYD6 regulated chemoresistance through mediating CRC cell apoptosis. (a) FXYD6 silenced cells and FXYD6 overexpressed cells were successfully constructed in SW620 and SW620/Iri cells. The expression level of FXYD6 was measured by RT-PCR. (b) MTT assay was carried out to confirm drug concentration of Iri and Oxa when the cell survival rate changed significantly compared to the nontreated group. (c) Flow cytometric analysis was performed in FXYD6 silenced SW620 cells and FXYD6 overexpressed SW620/Iri cells. The apoptosis rate was analyzed by GraphPad Prism 7. LR: early apoptosis; UR: late apoptosis. (d) Western blotting was performed on apoptosis element expression in FXYD6 silenced SW620 cells and FXYD6 overexpressed SW620/Iri cells. Relative abundance was analyzed by the ImageJ program.

**Figure 3:** FXYD6 regulated chemoresistance through mediating CRC cell autophagy. (a) SW620 and SW620/Iri cells stably expressed RFP (red puncta) after cotransfection. Autophagic puncta were documented by a fluorescence microscope (200x magnification). Scale bar: 20 *μ*m. Autophagic puncta were counted in 20 cells which were used to quantify. (b) Western blotting was conducted on autophagy elements in FXYD6 silenced and overexpressed cells, respectively. Relative abundance was analyzed by the ImageJ program; LC3I was the internal control of LC3II; *β*-actin was the internal control of Beclin1 and P62. (c) MTT assays were conducted to measure the cell survival rate when autophagy was activated or inhibited. Rapa is an autophagic stimulator, and 3-MA is an autophagic inhibitor; PBS and DMSO were used as the control group, respectively. (d) Flow cytometric analysis was used to test apoptosis when autophagy was activated with Rapa or inhibited with 3-MA. The apoptosis rate was analyzed by GraphPad Prism 7. LR: early apoptosis; UR: late apoptosis.

The article "FXYD6 Regulates Chemosensitivity by Mediating the Expression of Na+/K+-ATPase α1 and Affecting Cell Autophagy and Apoptosis in Colorectal Cancer" was retracted in 2024. Reasons: signs of a paper mill; compromised peer review; unreliable results or conclusions.

**Figure 4:** FXYD6 mediated cell apoptosis and autophagy by mediating the Na+/K+-ATPase *α*1 pathway in chemosensitivity regulation of CRC cells. (a) Protein expression of ATP-*α*1 in SW620/Iri and SW620 cells was documented by western blotting. Relative abundance was analyzed by the ImageJ program (upper). Relative expression of ATP-*α*1 in SW620/Iri and SW620 cells was detected by RT-PCR (lower). (b) Western blotting was conducted in FXYD6 and ATP-*α*1 silenced SW620 cells and FXYD6 and ATP-*α*1 overexpressed SW620/Iri cells to understand the relationship of FXYD6 and ATP-*α*1. Relative abundance was analyzed by the ImageJ program. (c) Western blotting was performed in ATP-*α*1 silenced cells built on SW620/Iri-FXYD6 cells and ATP-*α*1 overexpressed cells built on SW620-siFXYD6 cells. Relative abundance was analyzed by the ImageJ program. (d) Autophagy and apoptosis elements were tested by western blotting. LC3I was the internal control of LC3II; *β*-actin was the internal control of P62, BAX, and Bcl-2. (e) MTT assays were carried out to measure the cell survival rate. (f) The autophagy was documented under different expressions of ATP-*α*1 by autophagy fluorescence analysis using a fluorescence microscope (200x magnification). Scale bar: 20 *μ*m. Autophagic puncta were counted in 20 cells, and average puncta were used to quantify. (g) The apoptosis was tested by flow cytometric analysis under different expressions of ATP-*α*1. The apoptosis rate was analyzed by GraphPad Prism 7. LR: early apoptosis; UR: late apoptosis.

**Table 1:** Parameters of CRC patients (*n* = 5).

Number	Gender	Age (year)	pTNM staging
1	F	54	T_3_N_0_M_0_
2	F	67	T_2_N_0_M_0_
3	M	50	T_3_N_0_M_0_
4	F	65	T_3_N_0_M_0_
5	M	58	T_3_N_0_M_0_

**Table 2:** Details for primer sequences.

Primer names	Primer sequence
FXYD6-F	CTCTTCTCGGTTGGGATCCTC
FXYD6-R	GAAAGGGCTGTTGCTGAAGTG
ATP-*α*1-F	TTGGGCACTGACATGGTTCC
ATP-*α*1-R	TCAGCCGCTCATTCACAAGT
GAPDH-F	AGAAGGCTGGGGCTCATTTG
GAPDH-R	AGGGGCCATCCACAGTCTTC

The article "FXYD6 Regulates Chemosensitivity by Mediating the Expression of Na+/K+-ATPase α1 and Affecting Cell Autophagy and Apoptosis in Colorectal Cancer" was retracted in 2024. Reasons: signs of a paper mill; compromised peer review; unreliable results or conclusions.

**Table 3:** Details for interference sequences.

siRNA name	Sequence
siFXYD6	CUGGCAGGCAAUAGUUGAATT
siATP-*α*1	CUUGAUGAACUUCAUCGUAAA
siNC	UUCUCCGAACGUGUCACGUTT

**Table 4:** Details for the antibodies.

Reagents	Source	Identifier	Dilution
Anti-FXYD6	Proteintech	15805-1-AP	1 : 500
Anti-ATP-*α*1	Proteintech	14418-1-AP	1 : 500
Anti-LC3II/I	Cell Signaling Technology	4108S	1 : 1000
Anti-BAX	Cell Signaling Technology	2774S	1 : 1000
Anti-Bcl-2	Cell Signaling Technology	2875S	1 : 1000
Anti-Beclin1	Cell Signaling Technology	3738S	1 : 1000
Anti-*β*-actin	Cell Signaling Technology	4970S	1 : 1000

## Data Availability

The datasets used and/or analyzed during the present study are available from the corresponding author on reasonable request.
